# Effect of Left Atrial Appendage Closure in Combination With Catheter Ablation on Left Atrial Function for Persistent Atrial Fibrillation

**DOI:** 10.3389/fcvm.2021.666465

**Published:** 2021-04-30

**Authors:** Jing Yang, Yue Liu, Liang Feng, Mingqing Liu, Ling You, Yu Liu, Jinglan Wu, Guangming Zhang, Xue Geng, Ruiqin Xie

**Affiliations:** ^1^Division of Cardiology, The Second Hospital of Hebei Medical University, Shijiazhuang, China; ^2^Department of Medicine, Cangzhou Medical College, Cangzhou, China; ^3^Department of Cardiac Surgery, The Second Hospital of Hebei Medical University, Shijiazhuang, China

**Keywords:** left atrial appendage closure, catheter ablation, left atrial function, left atrial volumes, speckle tracking echocardiography

## Abstract

**Background:** A single procedure combining left atrial appendage closure (LAAC) plus catheter ablation (CA) has been proven to be safe and feasible for treating atrial fibrillation (AF). However, the influence of treatment modality on left atrial (LA) function is not thoroughly explained.

**Objective:** We aimed to investigate the changes of LA function in persistent AF patients undergoing concomitant LAAC and CA.

**Methods:** The study population comprised 65 patients who underwent combined AF ablation and Watchman LAAC (combined therapy group) in our center, and 65 participants of the AF simple ablation group who were matched based on sex, age, CHA_2_DS_2_-VASc score and HAS-BLED score using propensity score matching. During the 1-year follow-up period, two-dimensional echocardiography and speckle tracking echocardiography were performed to assess LA reservoir, conduit, and contractile function.

**Results:** The combined therapy was associated with a significant improvement in the LA reservoir function with increased expansion index and strain indices, including strain and strain rate (SR) during ventricular systole. Conduit function with SR during early ventricular diastole was also improved, as was contractile function with active atrial emptying fraction and SR during atrial systole. Similarly, LA reservoir and contractile function indices all improved continuously during follow-up after catheter ablation alone. At 3 months follow-up LA reservoir and conduit function with strain indices had a tendency to improve only in the simple procedure group. At 1-year follow-up there was no significant difference in either LA volumes or strain indices between the two groups.

**Conclusion:** Both the combined therapy group and the simple ablation group demonstrated significant improvement in LA function. Based upon the fact that LA function was improved in both groups it might be concluded that most of the effects appeared to result from ablation, not LAAC; furthermore the additional LAAC procedure did not affect the improvement of LA function after CA.

## Introduction

Atrial fibrillation (AF) is the most common type of cardiac arrhythmia and is a major cause of ischemic stroke worldwide. Catheter ablation is a safe and effective treatment for AF; however, long-term effects of this therapy remain unpredictable because arrhythmia recurs at high rates over time, especially in patients with persistent AF, who need ongoing stroke prevention treatment (1). In addition, research has confirmed that the CHA_2_DS_2_-VASc score (congestive heart failure, hypertension, age [>65 = 1 point, >75 = 2 points], diabetes mellitus, previous stroke or transient ischemic attack [2 points], vascular disease, and sex) is associated with prognosis of morbidity related to AF and inability in maintaining sinus rhythm after catheter ablation;(2) therefore, according to clinical practice guidelines, patients at high risk for stroke should continue long-term oral anticoagulation therapy, regardless of the outcome for heart rhythm.

The left atrial (LA) appendage is the main site of thrombus formation in patients with non-valvular AF. Closure of the left atrial appendage has been proposed as alternative to oral anticoagulation for stroke prophylaxis; studies have demonstrated that LAAC is as effective as warfarin and non–vitamin K oral anticoagulants in preventing strokes (3, 4). LAAC in combination with AF ablation in a single procedure, might be effective in both controlling sinus rhythm and preventing stroke, without the additional risk of multiple procedures (5, 6).

The LA appendage was previously considered a dormant embryological remnant. However, emerging evidence indicates that it is a functional organ that plays an important role in cardiac hemodynamics through its contractile properties, which are in fact greater and more consequential than those of the LA (7), contributing to LA compliance and function modulation (8, 9). Catheter ablation itself can also have an influence on LA function by restoring and maintaining sinus rhythm and iatrogenic myocardial damage. We consequently hypothesized that the combined therapy might play an important role in cardiac hemodynamics and affect LA function. Studies undertaken so far have provided inconsistent results about the effect of LA function after LAAC alone, and other studies have focused on the effect of combined therapy on LA size (10); however, the effect of this combination on LA function and the interaction between LAAC and CA has not been investigated. We examined the potential changes in LA volume, strain, and strain rate (SR) with the use of transthoracic and speckle tracking echocardiographies in patients with persistent AF. By comparing the echocardiographic changes between the combined therapy and simple ablation groups, the impact of the additional LAAC procedure on LA function after CA treatment was investigated. This may provide more insights into the selection of the best treatment strategy for LAAC management.

## Methods

### Study Population

This single-center study included 66 consecutive patients who underwent AF ablation and Watchman LAAC between April 2015 and October 2018. All the patients had persistent or long-standing persistent AF and underwent CA followed by LAAC at the Second Hospital of Hebei Medical University, Hebei, People's Republic of China. Persistent AF was defined as episodes lasting more than 7 days and long-standing persistent AF was defined as episodes lasting more than 12 months (11). The inclusion criteria were as follows: (1) aged ≥18 years; (2) symptomatic nonvalvular atrial fibrillation (NVAF) refractory to antiarrhythmic drugs; (3) one or more CHA2DS2-VASc risk factors; (4) high bleeding risk predicted by a HASBLED [Hypertension, Abnormal liver and renal function, Stroke, Bleeding history or predisposition, Labile international normalized ratio, Elderly age over 65 years and Drugs or alcohol intake] score ≥ 3 or previous major bleeding event during anticoagulation therapy; (5) preferred LAAC treatment as an alternative to long-term oral anticoagulants. The exclusion criteria were the occurrence of LA thrombus, significant valvular heart disease, an enlarged LA (≥55 mm) and additional ablation lines or CFAE ablation strategy. This study also included a control group comprising 174 participants with contemporaneous persistent AF who were undergoing AF ablation. The inclusion criteria were age ≥18 years and symptomatic NVAF refractory to antiarrhythmic drugs. The exclusion criteria were the same as those for the combined therapy group. Propensity score matching analysis (1:1 matching) using age, sex, CHA2DS2-VASc score, and HAS-BLED score was performed to control for selection bias within a caliper of 0.05 on the propensity-score using EmpowerStats software (http://www.empowerstats.com). Sixty-five patients were selected from each group. The study flowchart is shown in Figure 1. The study protocol was approved by the ethics committee of The Second Hospital of Hebei Medical University, in accordance with the ethical guidelines of the 1975 Declaration of Helsinki. Written consent was obtained from all the patients.

**Figure 1:** Flowchart of the study procedure. LA, left atrial; LAAC, left atrial appendage closure; CA, catheter ablation; AF, atrial fibrillation.

### Preprocedural Protocols

Transesophageal echocardiography and cardiac computed tomography were performed to rule out LA appendage thrombus and to evaluate the dimension and depth of the appendage before the procedure.

### Catheter Ablation Procedure

All procedures were performed while patients were under conscious sedation and local anesthesia. Pulmonary vein isolation (PVI) was performed in all cases with wide antral cricumferential until the entrance and exit block was demonstrated for each pulmonary vein. With a three-dimensional electroanatomical mapping system (CARTO®3; Biosense Webster, Irvine, CA, USA), the ablation catheter (Thermocool SMARTTOUCH; Biosense Webster) was inserted into the LA to perform radiofrequency ablation. The mapping catheter was used to record pulmonary vein potentials (Lasso® NAV Eco; Biosense Webster). Circumferential ablation was confirmed in both left and right pulmonary veins. No additional ablation lines or CFAE ablation was performed in this study. Sinus rhythm was restored by either ablation or electric cardioversion.

### Left Atrial Appendage Closure Procedure

In the combined therapy group, occluder devices for LA appendage were implanted under fluoroscopic or transesophageal echocardiographic guidance immediately after PVI. After catheter ablation, the LA appendage was occluded with the use of occluder devices (Watchman; Boston Scientific, Marlborough, MA, USA). The process of Watchman implantation is shown in Figure 2. Angiography of the LA appendage was performed to measure the ostial width and depth. Oversizing by 10–20% of the diameter of the LA appendage was recommended in order to choose an appropriate device size, and the device was released in the proper position after stability testing. Before releasing the occluder device, we ensured that no or minimal (<5 mm) residual flow remained and that adjacent structures (such as the mitral annulus and circumflex coronary artery) were not compressed.

**Figure 2:** Left atrial appendage closure with WATCHMAN device. **(A)** Left atrial appendage angiograph. **(B)** Ostial width and depth of LAA measured after angiograph. **(C)** Fluoroscopic view after delivery of the WATCHMAN device in the proper position. **(D)**: Peri-device leakage and compression were detected by TEE post-implantation.

### Echocardiographic Examination

Follow-up echocardiography at 1 week and 1, 3, 6, and 12 months after surgery was performed with a cardiac ultrasound device (iE33 system equipped with X3-1 probe; Philips Medical Systems, Eindhoven, The Netherlands). All patients had AF at baseline and were in sinus rhythm during follow-up examinations with comprehensive two-dimensional transthoracic echocardiography and speckle tracking echocardiography.

On two-dimensional transthoracic echocardiography, LA volumes were measured at three time points during the cardiac cycle: (1) at the end-diastolic frame before mitral valve opening (maximum LA volume [LAVmax]); (2) at the end-systolic frame before mitral valve closure (minimum LA volume [LAVmin]); and (3) at the time corresponding to the electrocardiographic P wave, or the last frame before the mitral valve opened (before atrial contraction [LAVpreA]) The process of LA volume measurements is shown in Figure 3.

**Figure 3:** LA function measured by LA volume and speckle tracking echocardiography. **(A)** Measurement of maximum LA volume, before atrial contraction LA volume and minimum LA volume. **(B)** Measurement of LA strain and strain rate in apical two- and four-chamber view. a,b Atrial strain and strain rate measured in apical four-chamber view. c,d Atrial strain and strain rate measured in apical two-chamber view.

LA mechanical function was derived from LA volumes and expressed in the following formulas (12):

Total atrial emptying fraction = [(LAVmax − LAVmin)/LAVmax] × 100%
Atrial expansion index (an index of LA reservoir function) = [(LAVmax − LAVmin)/LAVmin] × 100%
Passive atrial emptying fraction (an index of LA conduit function) = [(LAVmax − LAVpreA)/LAVmax] × 100%
Active atrial emptying fraction (an index of LA active contraction) = [(LAVpreA − LAVmin)/LAVpreA] × 100%

In addition, longitudinal LA wall deformation was assessed in apical views on speckle tracking echocardiography with cardiovascular ultrasound quantification software (QLAB Ultrasound Cardiac Analysis; Philips Medical Systems). In this novel software, motion is analyzed by tracking of the frame-to-frame movement of natural acoustic markers in two dimensions. The measurement method has been described in our previous work (13). LA strain, strain rate during ventricular systole (SRs), and strain rate during early ventricular diastole (SRe) were measured both during sinus rhythm and during AF. Strain rate during atrial systole (SRa) could only be measured during sinus rhythm, and so we summarized the trend of postoperative changes. The process of STE is shown in Figure 3.

### Arrhythmia Recurrence Assessment

All patients received antiarrhythmic drugs and anticoagulation regimens for 3 months postoperatively. If device-related thrombus or peri-device leaks ≥5 mm were not detected on TEE at 3 month, then the patients who underwent the combined therapy were recommended for another 3-month dual antiplatelet therapy (DAT; aspirin [100 mg od] plus clopidogrel [75 mg od]), and oral aspirin use was continued until 1 year postoperatively. Postprocedural 24-h monitor recordings were obtained 3, 6, and 12 months after surgery to evaluate the presence of atrial arrhythmias. AF or recurrent atrial flutter was defined as any documented AF or atrial flutter lasting more than 30 s after the blanking period without antiarrhythmic drug therapy.

### Statistical Analysis

Statistics were analyzed with SPSS Statistics, version 20 (IBM, Armonk, NY, USA). Kolmogorov–Smirnov test was applied to determine whether the data followed a normal distribution. Normally distributed data were expressed as mean ± standard deviation, while non-normally distributed data were shown as medians with interquartile ranges. Counting data were expressed as percentages (%). The student's *t*-test (normality) or Mann–Whitney *U* test (non-normality) and Chi-square test were used to compare the baseline parameters between the two groups of patients. Continuous data of different indices after the operation were assessed with analysis of variance for repeated measures. To compare LA function between the two groups, we used least significant difference test. A *p*-value of < 0.05 was considered statistically significant.

## Results

### Baseline Data

Of the 130 patients in this study, 65 underwent PVI alongside Watchman LAAC successfully (combined therapy group), and 65 matched controls underwent AF ablation only (simple ablation group). The clinical characteristics are reported in Table 1. All 130 patients had persistent AF, and long-standing persistent AF was present in 54% of combined therapy group and 46% of simple ablation group; the difference was not significant (*p* = 0.38). There was no significant difference in age or previous medical history between the two groups.

**Table 1:** Baseline characteristics of the population.

	**LAAC + CA**	**CA (*n* = 65)**	***p*-value**
	**(*n* = 65)**		
Age (years)	61.8 ± 7.9	60.7 ± 9.1	0.47
Sex male *n* (%)	40 (66)	43 (62)	0.72
Type of atrialfibrillation			0.38
Persistent AF *n* (%)	30 (46)	35 (54)	
Long-standing persistent AF *n* (%)	35 (54)	30 (46)	
Smoke *n* (%)	8 (12)	14 (21)	0.16
Alcohol *n* (%)	12 (18)	10 (15)	0.64
Labile INR *n* (%)	7 (11)	5 (8)	0.55
Hypertension *n* (%)	45 (69)	50 (77)	0.32
Coronary artery disease *n* (%)	15 (23)	12 (18)	0.52
Diabetes mellitus *n* (%)	9 (14)	10 (15)	0.80
Stroke *n* (%)	34 (52)	28 (43)	0.29
Bleeding *n* (%)	15 (23)	12 (18)	0.52
CHA2DS2- VASc score	3 (2, 4)	4 (3, 5)	0.09
HAS-BLED score	3 (2, 3)	3 (2, 3)	0.95

*Data are shown as mean ± SD or n (%)*.

*LAAC, left atrial appendage closure; CA, catheter ablation; AF, atrialfibrillation*.

### Left Atrial Function Assessed by Volumetric Indices

Out of the 130 patients, 45 were excluded due to sinus rhythm at baseline or AF or atrial flutter during follow-up echocardiography, leaving 85 patients (41 in combined therapy group and 44 in simple ablation group) for the analysis of LA volume, ƹ, and SR.

The patients in both the combined therapy and simple ablation groups showed significant decreases in left atrial diameter and LA volume. From baseline to 12 months after surgery, mean LA total emptying fraction increased from 31.8 ± 11.3 to 47.7 ± 12.5 (*p* < 0.001) in the combined therapy group and from 26.6 ± 13.0 to 50.8 ± 13.2 (*p* < 0.001) in the simple ablation group. LA reservoir function as assessed by expansion index improved significantly over time in both groups. The echocardiographic results indicated that from baseline to 12 months after surgery, the mean LA expansion index improved from 51.3 ± 29.6 to 102.2 ± 50.9 (*p* < 0.001) in the combined therapy group and from 41.0 ± 27.8 to 118.0 ± 60.7 (*p* < 0.001) in the simple ablation group. In addition, from 1 week to 12 months after surgery, mean active atrial emptying fraction, which in the LA reflects contractile function, increased significantly from 20.8 ± 13.5 to 32.1 ± 13.9 (*p* < 0.001) in the combined therapy group and from 24.9 ± 10.0 to 32.5 ± 12.3 (*p* = 0.014) in the simple ablation group. Of note, no significant changes were observed in LA conduit function, as assessed with passive atrial emptying fraction, at the 1-year follow-up visit in both groups. The results of the correlational analysis are listed in Table 2.

**Table 2:** Evolution of LA function after the LAAC combined with CA and simple CA group assessed volumetric indices.

	**Baseline**	**1 Week**	**1 Month**	**3 Months**	**6 Months**	**12 Months**	***F* value**	***p*-value**
Combined therapy group (*n* = 41)								
LAD	42.3 ± 4.0	41.3 ± 4.8	40.2 ± 4.1	39.1 ± 3.7	38.7 ± 3.6	38.5 ± 4.3	18.1	<0.001
LAV max (mL)	86.3 ± 15.5	82.2 ± 16.8	73.4 ± 18.5	72.2 ± 18.1	70.1 ± 19.3	71.1 ± 20.3	12.7	<0.001
LAV preA (mL)	–	62.0 ± 15.9	54.8 ± 17.3	54.5 ± 16.6	53.2 ± 18.1	55.4 ± 18.6	4.7	0.001
LAV min (mL)	59.6 ± 17.1	49.7 ± 17.1	43.2 ± 18.6	39.4 ± 15.1	38.2 ± 16.7	38.2 ± 16.5	24.7	<0.001
Total atrial EF	31.8 ± 11.3	40.9 ± 10.2	43.1 ± 13.4	46.3 ± 10.4	47.1 ± 11.5	47.7 ± 12.5	14.7	<0.001
Atrial expansion index	51.3 ± 29.6	74.4 ± 30.1	86.3 ± 49.0	92.5 ± 35.9	98.0 ± 44.5	102.2 ± 50.9	10.9	<0.001
Passive atrial EF	–	24.9 ± 9.0	26.0 ± 11.6	24.9 ± 9.0	25.0 ± 8.1	22.9 ± 9.2	0.6	0.597
Active atrial EF	–	20.8 ± 13.5	22.8 ± 15.8	28.5 ± 10.2	29.7 ± 11.7	32.1 ± 13.9	6.1	<0.001
Simple ablation group (n=44)								
LAD	40.9 ± 4.2	39.7 ± 4.3	38.7 ± 4.6	37.8 ± 4.1	39.9 ± 9.8	37.4 ± 3.6	3.8	0.039
LAV max (mL)	77.3 ± 21.1	71.1 ± 19.8	67.4 ± 20.5	69.1 ± 22.5	66.8 ± 19.8	68.3 ± 20.5	3.6	0.004
LAV preA (mL)	–	55.6 ± 16.9	53.0 ± 17.2	54.2 ± 19.8	51.9 ± 17.8	50.7 ± 19.1	1.8	0.132
LAV min (mL)	57.0 ± 19.7	42.4 ± 16.5	39.6 ± 17.4	38.9 ± 20.3	35.8 ± 16.9	34.2 ± 17.0	24.1	<0.001
Total atrial EF	26.6 ± 13.0	41.2 ± 10.8	42.9 ± 11.2	46.2 ± 10.6	48.5 ± 9.6	50.8 ± 13.2	24.8	<0.001
Atrial expansion index	41.0 ± 27.8	77.1 ± 42.8	81.4 ± 34.2	92.4 ± 35.3	101.1 ± 39.0	118.0 ± 60.7	16.4	<0.001
Passive atrial EF	–	21.4 ± 12.0	21.4 ± 10.3	22.0 ± 9.9	23.1 ± 9.9	27.0 ± 12.9	2.4	0.054
Active atrial EF	–	24.9 ± 10.0	26.4 ± 14.6	30.4 ± 13.5	32.8 ± 11.3	32.5 ± 12.3	3.8	0.014

*Data are shown as mean ± SD*.

*LAD, left atrialdiameter; LAV, left atrial volume; EF, emptying fraction*.

Comparisons of the LA diameter volumes and function in the two groups as assessed by volumetric indices are shown in Figure 4. During the 1-year follow-up visit, we found no significant differences between the two groups in left atrial diameter or in LA volumetric indices, including LA volumes, LA total emptying fraction, expansion index, passive emptying fraction, and active emptying fraction.

**Figure 4:** Comparisons of the LA diameter volumes and function in the two groups as assessed by volumetric indices. **(A)** Comparison of left atrial diameter (LAD) and volume (LAV) between the combined therapy group (Group 1) and those who underwent simple ablation group (Group 2). **(B)** Comparison of atrial function, as assessed by volumetric indices, between the two groups. We found no differences in left atrial diameters, left atrial volumes, left atrial total emptying fractions, expansion indices, or passive or active emptying fractions. Variables are expressed as means ± standard deviations. *p < 0.05 vs. the combined therapy group at the same follow-up time.

### Left Atrial Function Assessed by Strain Indices

The combined therapy was associated with a significant improvement in LA reservoir function and in strain indices including strain and SRs in echocardiographic views of two chambers (strain: from 15.0 ± 4.0 to 29.1 ± 7.5, *p* < 0.001; SRs: from 1.0 ± 0.4 to 1.7 ± 0.5, *p* < 0.001) and four chambers (strain: from 16.5 ± 7.1 to 29.4 ± 8.9, *p* < 0.001; SRs: from 1.0 ± 0.4 to 1.6 ± 0.5, *p* < 0.001). It also resulted in improved conduit function with SRe in the two-chamber (from −1.5 ± 0.5 to −1.7 ± 0.5, *p* < 0.001) and four-chamber views (from −1.4 ± 0.6 to −1.8 ± 0.6, *p* < 0.001) and in improved contractile function with SRa in two-chamber (from −1.2 ± 0.6 to −2.0 ± 0.7, *p* < 0.001) and four-chamber views (from −1.2 ± 0.6 to −2.0 ± 0.7, *p* < 0.001). Similarly, in the simple ablation group, strain indices in LA reservoir function showed significant improvement in two-chamber (strain: from 16.5 ± 7.0 to 31.8 ± 10.4, *p* < 0.001; SRs: from 0.9 ± 0.3 to 1.7 ± 0.4, *p* < 0.001) and four-chamber views (strain: from 18.0 ± 7.4 to 32.1 ± 10.5, *p* < 0.001; SRs: from 1.0 ± 0.4 to 1.6 ± 0.6, *p* < 0.001), as did contractile function in two-chamber (from −1.4 ± 0.5 to −2.0 ± 0.9, *p* = 0.003) and four-chamber views (from −1.2 ± 0.6 to −2.0 ± 0.9, *p* < 0.001). In addition, the simple ablation group showed no statistically significant change in conduit function with SRe in two-chamber (from −1.6 ± 0.7 to −1.6 ± 0.7, *p* = 0.617) and four-chamber views (from −1.6 ± 0.7 to −1.7 ± 0.7, *p* = 0.076). The results obtained from the preliminary analysis of LA strain and SR are displayed in Table 3.

**Table 3:** Evolution of LA function after the LAAC combined with CA and simple CA group assessed strain indices.

	**Baseline**	**1 Week**	**1 Month**	**3 Months**	**6 Months**	**12 Months**	***F* value**	***p*-value**
Combined therapy group (*n* = 41)								
ƹ (2-chamber)	15.0 ± 4.0	20.7 ± 8.7	23.2 ± 6.4	25.9 ± 9.8	28.5 ± 8.3	29.1 ± 7.5	34.7	<0.001
ƹ (4-chamber)	16.5 ± 7.1	20.1 ± 7.8	24.0 ± 7.6	26.9 ± 8.8	28.9 ± 9.1	29.4 ± 8.9	33.9	<0.001
SRs (2-chamber)	1.0 ± 0.4	1.2 ± 0.5	1.4 ± 0.4	1.3 ± 0.6	1.6 ± 0.4	1.7 ± 0.5	16.7	<0.001
SRs (4-chamber)	1.0 ± 0.4	1.1 ± 0.3	1.3 ± 0.4	1.4 ± 0.4	1.6 ± 0.4	1.6 ± 0.5	25.5	<0.001
SRe (2-chamber)	−1.5 ± 0.5	−1.3 ± 0.5	−1.4 ± 0.4	−1.4 ± 0.5	−1.6 ± 0.5	−1.7 ± 0.5	10.2	<0.001
SRe (4-chamber)	−1.4 ± 0.6	−1.4 ± 0.5	−1.4 ± 0.5	−1.5 ± 0.5	−1.6 ± 0.6	−1.8 ± 0.6	9.1	<0.001
SRa (2-chamber)	–	−1.2 ± 0.6	−1.5 ± 0.6	−1.7 ± 0.7	−1.9 ± 0.7	−2.0 ± 0.7	24.1	<0.001
SRa (4-chamber)	–	−1.2 ± 0.6	−1.5 ± 0.6	−1.6 ± 0.6	−1.9 ± 0.8	−1.9 ± 0.7	23.3	<0.001
Simple ablation group (n=44)								
ƹ (2-chamber)	16.5 ± 7.0	24.6 ± 7.9	30.0 ± 9.1	32.0 ± 11.6	31.7 ± 11.2	31.8 ± 10.4	37.1	<0.001
ƹ (4-chamber)	18.0 ± 7.4	25.8 ± 8.2	28.4 ± 10.3	31.4 ± 10.5	32.5 ± 9.8	32.1 ± 10.5	25.6	<0.001
SRs (2-chamber)	0.9 ± 0.3	1.4 ± 0.5	1.7 ± 0.8	1.6 ± 0.6	1.7 ± 0.6	1.7 ± 0.4	16.4	<0.001
SRs (4-chamber)	1.0 ± 0.4	1.3 ± 0.4	1.5 ± 0.5	1.6 ± 0.6	1.6 ± 0.5	1.6 ± 0.6	18.7	<0.001
SRe (2-chamber)	−1.6 ± 0.7	−1.6 ± 0.7	−1.7 ± 0.7	−1.7 ± 0.7	−1.6 ± 0.6	−1.6 ± 0.7	0.7	0.617
SRe (4-chamber)	−1.6 ± 0.7	−1.6 ± 0.5	−1.7 ± 0.6	−1.8 ± 0.6	−1.8 ± 0.7	−1.7 ± 0.7	2.0	0.076
SRa (2-chamber)	–	−1.4 ± 0.5	−1.9 ± 0.9	−1.8 ± 1.3	−2.0 ± 0.8	−2.0 ± 0.9	5.3	0.003
SRa (4-chamber)	–	−1.2 ± 0.3	−1.6 ± 0.8	−1.8 ± 1.1	−1.8 ± 1.0	−2.0 ± 0.9	10.2	<0.001

*Data are shown as mean ± SD*.

*ƹ, strain; SR, strain rate; SRs, strain rate during ventricular systole; SRe, strain rate during early ventricular diastole; SRa, strain rate during atrial systole*.

At 3 months follow-up LA reservoir and conduit function with strain indices had a tendency to improve only in the simple procedure group. At 1-year follow-up there was no significant difference in strain indices between the two groups. Figure 5 shows comparisons of LA function as assessed by strain indices between the two groups in both two- and four-chamber views.

**Figure 5:** Comparison of left atrial function between the two groups as assessed by strain indices, in echocardiographic views of two chambers **(A)** and four chambers **(B)**. All the strain indices had a transient tendency to improve in the patients who underwent catheter ablation alone and the difference between the two groups began very early, between 1 week and 3 months after surgery. However, between months 6 and 12 after surgery, left atrial (LA) function was not significantly different between the two groups. Group 1 consisted of combined therapy group; group 2 consisted of patients who underwent catheter ablation alone. Variables are expressed as means ± standard deviations. SR, strain rate; SRs, strain rate during ventricular systole; SRe, strain rate during early ventricular diastole; SRa, strain rate during atrial systole. *p < 0.05 vs. the combined therapy group at the same follow-up time.

### Clinical Outcome

Pulmonary veins were isolated and sinus rhythm was restored in all patients. During the 12 months of follow-up, 18 patients (28%) in combined therapy group and 16 patients (25%) in simple ablation group had recurrent AF or atrial flutter (*p* = 0.69). In the combined therapy group, all procedures were successful, and all implants were satisfactorily sealed (residual leak <5 mm). One patient had pericardial effusion and required percutaneous drainage. Acute left-sided heart failure occurred in one patient 2 days after the hybrid procedure as a result of postoperative rehydration; diuretic treatment was provided immediately. Device-related thrombus was observed in one patient, and no peri-device leaks ≥5 mm were detected at the 3-month TEE follow-up. During the 12 months of follow-up, no patients exhibited device dislocation, thromboembolic events, or ischemic stroke. One major bleeding events (severe intracerebral hemorrhage in a patients treated with rivaroxaban at 2 months) and one minor bleeding events (epistaxis in a patients treated with with dual anti-platelet therapy at 6 months) were observed, with no hemorrhagic deaths reported. In the simple ablation group, one patient developed a groin hematoma 2 days postoperatively, and one had a cerebral hemorrhage 3 months after the AF ablation, which was resolved with conservative treatment.

## Discussion

The major findings of our study are as follows: (1) Both the combined therapy group and the simple ablation group demonstrated significant improvement in LA function on echocardiography at the 12-month follow-up visit. (2) Hemodynamic effects were substantially different between LAAC with endocardial devices combined with catheter ablation and catheter ablation alone at the 3-month follow-up; however, the LA function in the two groups did not differ significantly at the 6-month and 1-year follow-up visits. (3) Even though LA function was improved by the combined therapy, most of the effects appeared to result from ablation, but not LAAC. These results suggest that the additional LAAC procedure did not affect the improvement of LA function after CA.

Normal LA function can be divided into three distinct phases. During ventricular systole, the LA serves as a reservoir for blood drained by the pulmonary veins. LA reservoir function reflects the ability of the LA to store pulmonary venous return during left ventricular contraction and isovolumetric relaxation. During early ventricular diastole, the LA is a conduit for the pulmonary venous return. Conduit LA function reflects the ability to passively transfer blood into the left ventricle. During late diastole, the contractile function of the LA completes left ventricular filling during the last diastolic phase (14, 15).

In our study, echocardiography results indicated that LA function was improved both in patients undergoing combined therapy and in those undergoing catheter ablation alone, and did not differ significantly between the two groups at the 1-year follow-up visit. Based upon the fact that LA function was improved in both groups it might be concluded that most of the effects appeared to result from ablation, not LAAC. Previous studies demonstrated that persistent AF ablation was associated with a dramatic improvement in mechanical cardiac functions, and this evidence further supports our inference (16, 17).

Moreover, simple CA can achieve better improvement of LA function as compared to the combined therapy before 3 months, and the difference between the two groups in LA reservoir and conduit function as assessed by strain indices began very early, from 1 week to 3 months after surgery. However, between months 6 and 12, LA function did not differ significantly between the two groups. These findings indicate that performing LAAC as a concomitant procedure to CA did not translate into any significant changes in LA contractive function, but it may result in a transient decline in left atrial reservoir and conduit function.

The left atrial appendage is a blind pouch-like structure arising from the LA and plays an important role in cardiac hemodynamic function through its contractile properties. Several lines of evidence suggest that the left atrial appendage is more compliant than the LA main chamber and that LA compliance decreases after removal of the left atrial appendage (8, 9, 18). Endocardial occlusion devices formed mostly a mechanical barrier between the left atrial appendage and the LA and could cause a decline in atrial compliance. However, both the LA reservoir and conduit functions are influenced by LA compliance (14), and this may be the reason why additional LAAC is characterized by a transient decrease in LA reservoir and conduit function. After the 6-month follow-up visits, the two groups showed no statistical difference in LA function, which implied that after a period of adaptation, LA function gradually recovered and eventually became equivalent to that in the control group.

To date, the role of LAAC in LA function has been controversial. Previous studies have demonstrated that percutaneous LAAC did not translate into any significant changes in LA function as assessed by LA volume and strain indices (19, 20). The same results were also reported in patients with surgical LA appendage exclusion (21), which is consistent with our findings. However, different conclusions were drawn in other studies. Coisne et al. (22) reported that LAAC was associated with an improvement in LA mechanical function through the Frank-Starling mechanism, and these results were reinforced by similar results obtained in patients who underwent LA appendage exclusion by epicardial ligation (23).

The heterogeneity of the results may be related to the differences in the study populations, in indicators representing LA function and the length of follow-up. Previous studies have shown that flow pattern and flow velocity in the LA appendage during AF differ from those during sinus rhythm (7). Therefore, different types of AF differentially affect hemodynamic function after LAAC, and this might be the main reason for the inconsistent results of previous studies. In addition to this, different indicators might affect the results and lead to inconsistent findings.

Our findings have important implications for future research and clinical practice. The impact of LAAC on the rhythm outcomes of AF ablation is still not clear. Our results showed that the AF recurrence rate of the combined group was comparable with that of the CA-only group during 1 years follow-up, indicating that additional LAAC did not influence the recurrence rate of atrial fibrillation. This finding is in line with previous literature (24, 25). Moreover, Persistent AF, even long-standing persistent AF, is difficult to treat inasmuch as arrhythmia recurs at significant rates after catheter ablation therapy. Hence, this study focuses on patients with persistent AF at high risk of stroke and bleeding and further examines optimized therapeutic strategies. Research shows that the combined therapy may be a cost-effective therapeutic option compared with CA therapy for symptomatic AF patients with high risks of stroke and bleeding (26). It is well-known that treatment with AF ablation can substantially improve cardiac function; however, the effects of LAAC on cardiac function is somewhat controversial, and the best treatment strategy for LAAC management is remains debatable. Despite the evidence supporting the significant increase in LAV after LAAC (27, 28). LA structural reverse remodeling could be evidenced in patients after the combined therapy (10). In this study, we obtained the same results. Additionally, the present study also demonstrates that combined therapy significantly improved LA function; however, CA alone can achieve better improvement of cardiac function compared with the combined therapy before 3 months. These results suggest that rhythm control plays a prominent role in improving LA function, which outweighs the transient detrimental effects of LAAC. Therefore, the combination of LAAC and catheter ablation may be a valuable and practical approach to restoring and maintaining sinus rhythm and preventing stroke. The additional LAAC procedure did not affect the improvement of LA function after CA.

### Limitations

Several limitations in this study must be acknowledged. The sample size was small, and we lacked a group of patients who underwent LAAC alone, which would have served as historical control to indicate whether LAAC had an effect on LA function. Of the patients at our institution who underwent LAAC treatment alone, all were in AF both at baseline and during the follow-up period. Heart rhythms differed among the participants; therefore, analyzing the echocardiographic data during follow-up would have been difficult if the study had included a group that underwent LAAC only. Notwithstanding the relatively small sample, however, this study offers novel, valuable insights into the change in LA function after combined therapy.

The retrospective nature of the study was another limitation. Further prospective studies are needed to fully delineate the effect of the combined procedure on LA function.

## Conclusion

LA function was improved in the patients who underwent combined therapy and those who received CA therapy alone. Based upon the fact that LA function was improved in both groups it might be concluded that most of the effects appeared to result from ablation, not LAAC; furthermore the additional LAAC procedure did not affect the improvement of LA function after CA.

## Data Availability Statement

The datasets generated for this article are not readily available because The datasets generated and/or analyzed during the current study are not publicly available but are available from the corresponding author on reasonable request. Requests to access the datasets should be directed to Ruiqin Xie xieruiqin66@163.com.

## Ethics Statement

The studies involving human participants were reviewed and approved by Research Ethics committee of the second hospital of Hebei medical university. The patients/participants provided their written informed consent to participate in this study.

## Author Contributions

All authors listed have made a substantial, direct and intellectual contribution to the work, and approved it for publication.

## Conflict of Interest

The authors declare that the research was conducted in the absence of any commercial or financial relationships that could be construed as a potential conflict of interest.
